This article has been retracted.

# TGF-β2 initiates autophagy via Smad and non-Smad pathway to promote glioma cells’ invasion

**DOI:** 10.1186/s13046-017-0628-8

**Published:** 2017-11-16

**Authors:** Chao Zhang, Xin Zhang, Ran Xu, Bin Huang, An-Jing Chen, Chao Li, Jian Wang, Xin-Gang Li

**Affiliations:** 1 Department of Neurosurgery, Qilu Hospital of Shandong University, 107 Wenhua Western Rd, Jinan, Shandong 250012 China; 2 Brain Science Research Institute, Shandong University, 44 Wenhuaxi Road, Jinan, China; 3 Department of Biomedicine, University of Bergen, Bergen, Norway

**Keywords:** Malignant brain tumor, Autophagy, TGF-β, Tumor invasion, Galunisertib

## Abstract

**Background:**

Glioblastoma multiforme (GBM) is characterized by lethal aggressiveness and patients with GBM are in urgent need for new therapeutic avenues to improve quality of life. Current studies on tumor invasion focused on roles of cytokines in tumor microenvironment and numerous evidence suggests that TGF-β2 is abundant in glioma microenvironment and vital for glioma invasion. Autopagy is also emerging as a critical factor in aggressive behaviors of cancer cells; however, the relationship between TGF-β2 and autophagy in glioma has been poorly understood.

**Methods:**

U251, T98 and U87 GBM cell lines as well as GBM cells from a primary human specimen were used in vitro and in vivo to evaluate the effect of TGF-β2 on autophagy. Western blot, qPCR, immunofluorescence and transmission-electron microscope were used to detect target molecular expression. Lentivirus and siRNA vehicle were introduced to establish cell lines, as well as mitotracker and seahorse experiment to study the metabolic process in glioma. Preclinical therapeutic efficacy was evaluated in orthotopic xenograft mouse models.

**Results:**

Here we demonstrated that TGF-β2 activated autophagy in human glioma cell lines and knockdown of Smad2 or inhibition of c-Jun NH2-terminal kinase, attenuated TGF-β2-induced autophagy. TGF-β2-induced autophagy is important for glioma invasion due to the alteration of epithelial-mesenchymal transition and metabolism conversion, particularly influencing mitochondria trafficking and membrane potential (△Ψm). Autopaghy also initiated a feedback on TGF-β2 in glioma by keeping its autocrine loop and affecting Smad2/3/7 expression. A xenograft model provided additional confirmation on combination of TGF-β inhibitor (Galunisertib) and autophagy inhibitor (CQ) to better “turn off” tumor growth.

**Conclusion:**

Our findings elucidated a potential mechanism of autophagy-associated glioma invasion that TGF-β2 could initiate autophagy via Smad and non-Smad pathway to promote glioma cells’ invasion.

**Electronic supplementary material:**

The online version of this article (10.1186/s13046-017-0628-8) contains supplementary material, which is available to authorized users.

## Background

Malignant brain tumors are among the most intractable tumors and are known for their devastating proliferation, invasion and chemotherapy resistance [1]. Despite enormous efforts to target various pathways by suppressing oncogenes or angiogenesis, no improvement in survival has occurred, necessitating further study of the mechanisms of glioma oncogenesis [2]. Of all the hallmarks of glioma, the invasive ability poses a great barrier to surgeons and limits treatment options. Survival is measured in months (median survival is 14.6 months) [3]. In aggressive tumors, many kinds of autocrine and paracrine cytokines derived from astrocytes, microglia or glioma were found, which promotes tumor cell invasion, progression and metastasis. And during glioma invasion, the cytokines are reported to promote the trans-differentiation of immobile, polarized epithelial cells to motile, invasive mesenchymal cells, which is known as the epithelial-mesenchymal transition (EMT) [4–6]. Thus, much research has focused on the effect of cytokines on glioma invasion [7, 8].

Among the cytokines, TGF-β (transforming growth factor-β) is reported to be associated with essential molecules in glioma invasion [9–11]. And also in high grade tumors, increased TGF-β is related with poor clinical prognosis [8, 12, 13]. TGF-β could be divided into three isoforms in mammals: TGF-β1, TGF-β2, TGF-β3 and shared approximately 80% amino acid sequence identity and are distributed in different tissues [14].

In all the isoforms of TGF-β, TGF-β2 is specifically overexpressed in highly aggressive glioma and is involved in brain tumor development [14, 15]. Elevated TGF-β2 expression levels are usually observed in the later stages of tumor progression and in up to 95% of high grade gliomas [15–17]. TGF-β2 initiates an autocrine loop to promote its own expression and enable oncogenic activity. Thus the hyperactive TGF-β pathway and its key role in glioma oncogenesis provide a new target to cure gliomas. For instance, the TGF-β pathway inhibitors AP12009 and Galunisertib have been applied in phase II/III clinical cases, yielding encouraging results [18, 19].

Besides, this cytokine also has a dual role in oncogenesis. Depending on conditions and tumor stage, TGF-β can act as either a tumor suppressor or as a tumor promoter [19, 20].The mechanism of TGF-β transformation from tumor suppressor to tumor promoter is unclear. Currently, researchers are searching for the “switch factors” causing this behavior.

Previous studies have shown that autophagy could be activated by TGF-β and potentiate TGF-β-mediated growth inhibition in human hepatocellular carcinoma cells [21]. In our experiments, we tried to elucidate the effect of TGF-β on glioma from the autophagy aspect. Autophagy is an evolutionarily conserved lysosomal degradation pathway in which the cell re-digests its own proteins and organelles, thus maintaining macromolecular synthesis and ATP production [22]. The intactness of this flux is important for tumor cell invasion which consumes high levels of ATP, involves secretion factors, and reorganizes skeleton proteins [23, 24]. The inhibition of autophagy impairs tumor cell invasion. [25] Autophagy-mediated tumor promotion may work through suppressing the p53 response, maintaining mitochondria function, sustaining metabolic homeostasis and preventing the diversion of tumor progression [26]. However, the exact mechanism underlying how autophagy impairs glioma tumor progression needs to be explored and relationship between autophagy and cytokines also needs large studies. As autophagy and TGF-β are both involved in glioma invasion and participate in similar tumor functions, whether there are innate connections between these two factors in glioma and whether these associations influence glioma oncogenesis remain unknown. Our current study reports that TGF-β2 activates autophagy in glioma, influencing glioma invasion and metabolism reprogramming.

## Methods

### Cell culture and reagents

The high-grade, human glioma cell lines U251, U87 MG and T98G were obtained from American Type Culture Collection (Manassas, VA, USA) and used for in vitro experiments. Tumor cells were maintained as monolayer cultures in Dulbecco’s Modified Eagle’s Medium (DMEM; GIBCO) supplemented with 5% fetal calf serum (FCS). Primary cell line (P3) was obtained from the Department of Biomedicine, University of Bergen. When indicated, the cells were treated with TGF-β2 (10 ng/ml; PeproTech) and/or the small molecule TGF-β receptor inhibitor LY2157299 (10 μM; Selleck), chloroquine (10 μM; Selleck), bafilomycin A1 (10 μM; Tocris) and rapamycin (20 μM; Selleck). The inhibitor was added 2 h before the addition of TGF-β2.

### Constructs, transfection, and lentiviral/retroviral infection

The siATG5, siATG7 shRNA-expressing vector was obtained from GenePharma (Shanghai, China). GFP-LC3 (pBABEpuro, 22,405)-expressing vectors were obtained from Addgene (Cambridge, MA, USA). For the stable downregulation of ATG5, ATG7 scrambled and shRNA pGIPZ vectors were purchased from Open Biosystems (Thermo Scientific) or obtained through the Open Biosystems library. Lentiviral and retroviral supernatants were prepared following the manufacturer’s instructions and provided by GenePharma. Lentiviral infections were carried out accordingly. A validated Stealth RNAi (GenePharma) specific to Smad2 was also transfected into the U251, T98, and U87 cells using Lipofectamine 2000 according to the manufacturer’s protocol.

### Migration and invasion assays

The migratory ability of cells was determined by wound healing assays. The rate of wound closure was monitored at different time points under a microscope and quantified using ImageJ software. The invasion potential was determined on collagen coated Transwell assay (Corning, 8um). DMEM containing 0.1% FBS was added to the upper wells, while DMEM containing 10% FBS (a chemoattractant) was added to the lower wells. Transwell insert membranes were fixed and then stained with 0.25% eosin. Representative pictures of the membranes with cells were acquired at 40× magnification, and the total number of cells in 10 individual fields per membrane were counted.

### Western blotting

In brief, the cells were harvested, and lysed with protein extraction agent (Beyotime, Beijing, China). 25–50 μg of proteins per sample per lane were loaded for sodium dodecyl sulfate-polyacrylamide gel electrophoresis (SDS-PAGE). Primary antibodies were incubated overnight at 4 °C. Rabbit polyclonal primary antibodies were used against LC3B, SQSTM1, MMP2, MMP9, vimentin, N-cadherin, β-catenin, Slug2, Akt, JNK, SMAD2 (1:1000; Cell Signaling), TGF-β2 (1:500; Abcam), phospho-SMAD2, phospho-Akt, and phospho-JNK (1:500; Cell Signaling). Purified mouse anti-β-actin was used (1:1000; Santa Cruz Biotechnology, Inc.). Secondary antibodies were incubated with anti-mouse immunoglobulin G (IgG), anti-rabbit IgG (1:5000; Santa Cruz Biotechnology) for 1 h at RT. The proteins were visualized using Millipore’s enhanced chemiluminescence (ECL) and detection system analyzed (ChemiDoc Touch, BioRad).

### Intracranial injection mouse model

U87 cells were prepared for intracranial injection into NOD SCID male mice obtained from Vital River Laboratories. A total of five animals per condition were used, and animals were grouped as follows: PBS group, LY2157299 (75 mg/kg/d) group, CQ (25 mg/kg/d) group and LY2157299 (75 mg/kg/d) combined with CQ (25 mg/kg/d) group, drugs were used by oral application and 10ul U87 cells (1 × 10^6^/μl PBS) were injected in the cerebral cortex using a stereotactic frame. The mice were monitored and killed when they presented with neurological signs or after two months, during which time the tumor volumes and invading distance were monitored by MRI (General Electric, 3.0 T). Brains of three groups (PBS group, LY2157299 group and LY2157299 combined CQ group) were harvested and fixed in 4% paraformaldehyde for 48 h, embedded in paraffin and prepared for IHC. These experiments were approved by the Animal Care and Use Committee of Shandong University and conformed to the Animal Management Rule of the Chinese Ministry of Health (documentation 55, 2001).

### Quantitative real-time PCR

Total RNA was isolated using the RNeasy mini kit (Qiagen) according to the manufacturer’s instructions. RNA was analyzed quantitatively using a Nanodrop (Nanodrop Technologies, Rockland, DE, USA). Total RNA (1 μg) was reverse transcribed into cDNA using a cDNA synthesis kit (Toyobo) according to the manufacturer’s instructions. RT-PCR was performed in a Roche LightCycler 2.0 detector with the Toyobo SYBR Green Supermix. The reactions were analyzed using SDS software (Version 2.4). The threshold cycles (CT) were calculated and the relative gene expression was analyzed after normalizing to glyceraldehyde 3-phosphate dehydrogenase (GAPDH). The human primers are listed in Additional file 1: Figure S1.

### Immunofluorescence

GBM cells were plated on glass slides in 24-well culture plates at a concentration of 2 × 10^5^ cells/well for 24 h and were subsequently treated with drugs for an additional 48 h in DMEM containing FBS. The cells were then fixed with a 4% formaldehyde solution in PBS, permeabilized with 0.5% Triton X-100 in PBS, stained with primary antibody overnight, and labeled with anti-mouse or anti-rabbit IgG conjugated with FITC and DyLight 594 (Santa Cruz Biotechnology). The cells were counterstained with DAPI and observed under an Olympus BX61 fluorescence microscope. Pictures were scanned using a DP71 CCD (charge-coupled device) digital camera.

### Mitochondrial morphology

Live cells were fluorescently labeled with 25 nM MitoTracker Red (Invitrogen, Molecular Probes) and were then fixed and permeabilized for antibody conjugating. All treatments were performed according to the manufacturer’s instructions. Mitochondrial morphology was analyzed using an Olympus BX61 fluorescence microscope.

### Measurement of △Ψm

For the △Ψm measurements, the cells were loaded with 50 nM tetramethylrhodamine methylester (JC-1) for 30 min at room temperature. The dye was present during the experiment according to the manufacturer. The mitochondrial membrane potential was analyzed using an Olympus BX61 fluorescence microscope equipped with a 40× objective and quantified by flow cytometry (Novocyte, ACEA).

### Enzyme-linked Immunosorbent assay

For the quantitative determination of activated human TGF-β2, MMP2, MMP9 concentrations in cell culture supernatants, the quantitative sandwich enzyme immunoassay technique was used with commercially available, specific immunoassay kits for human TGF-β2 (R&D Systems), MMP2, and MMP9 (eBioscience). The minimum detectable dose of TGF-β2 was less than 7.0 pg/ml. The assay was performed in triplicate according to the manufacturer’s instructions.

### ATP—Lactate determination

The total ATP and lactate levels were measured by plating 2 × 10^5^ cells in 6-well plates overnight. The ells were counted and media samples were collected for ATP and lactate assays. The total ATP levels were determined using the Cell Titer-Glo Luminescent assay (Promega) according to the manufacturer’s instructions. Lactate was measured using the L-Lactate assay kit (Abcam). The data were expressed as moles of ATP and mg/dl lactate, and all values were normalized to the number of cells.

### Statistical analysis

Results are presented as the mean ± SD from at least three independent experiments. The comparisons were performed using with two-tailed Student’s t test, Spearman correlation test, Pearson correlation test, Wilcoxon matched-pair test, one-way ANOVA and long-rank analyse. Significant differences: *p < 0.05; **p < 0.01;***p < 0.001.

## Results

### TGF-β2 and LC3B are highly expressed in glioma and correlated with each other indicating poor prognosis in glioma patients

Although large studies has been conducted [27, 28], the role of autophagy’s markers Light Chain 3B (LC3B), ATG5 and ATG7 in glioma prognosis was still controversial. By applying immunochemistry on samples with different pathologic grades obtained from patients in Qilu Hospital, China from 2012 to 2015, we found that the percentage of LC3B, ATG5, ATG7 positive cells was associated with the pathologic grade (Fig. 1a). During this IHC process, we also found abundant TGF-β2 positive cells in GBM samples accompanied with autophagy markers positive. To quantitatively analyze the immunochemistry samples, we used the IRS scoring model (IRS = SI (staining intensity) × PP (percentage of positive cells)) [29], Wilcoxon matched-pair test, and Spearman correlation test to assess the results. Then the autophagy related markers and TGF-β2 were both identified to be associated with the pathologic grades (Fig. 1b) and correlated with each other when searched in REMBRANDT database (Fig. 1c).

**Fig. 1:** TGF-β2 and LC3B are highly expressed in glioma and co-localized with each other indicating poor prognosis in glioma patients. **a** Immunochemistry (IHC) showed more LC3B and TGF-β2 positive cells in GBM than normal brain (scale bars, 100μm). **b** IRS model quantatively analyzed LC3B and TGF-β2 expression levels in IHC and the correlationship between the two factors. **c** Relationship between TGF-β2 and autophagy related factors were calculated with Pearson index by data from REMBRANDT. **d** Immunofluorescent analysis of LC3B (green) and (red) co-localization in glioma and normal brain tissue (scale bars, 200μm, enlarged 50μm). **e** qRT-PCR analyses were compared between normal brain and glioma patients. **f** Chi-square analysis of age, gender or LC3B/TGF-β2 expression levels with glioma grades. **g** Long-rank monovariate analysis test in 63 glioma patients. **h** Survival curve about patients with TGF-β (+)/TGF-β (-) and TGF-β (+)/LC3B (+) were distinguished from TGF-β (+)/LC3B (-)

To further explore the relationship between autophagy and TGF-β, we concentrated on LC3B and TGF-β.The immunofluorescence images indicated that these two molecules were co-localized in glioma tissues (Fig. 1d). We verified these conclusions in primary tumor samples and qRT-PCR analysis showed similar results in normal brain tissues and glioma patients: Student’s t test, LC3B: GBM vs Normal, *p* = 0.0401, TGF-β2: GBM vs Normal, *P* = 0.0490; Pearson correlation test, *r* = 0.4101, *p* = 0.0144 (Fig. 1e).

Then based on the data we obtained from qRT-PCR, LC3B and TGF-β2 expression levels were also found to be associated with glioma grades in Chi-square test, whereas patient age and gender had no influence (Fig. 1f). We then added the survival time index and used the long-rank test to analyze. Data showed that high TGF-β2 expression indicated poor prognosis and short survival time in glioma patients (Fig. 1g). And among the samples with high TGF-β2 expression, robustly positive LC3B expression usually indicated a worse survival outcome (Fig. 1h). As the relationship between TGF-β2 and autophagy in glioma has not been explored, these results indicate that TGF-β2 and LC3B are highly expressed in glioma and correlated with each other. High expression levels of TGF-β2 with LC3B indicates poor prognoses in glioma patients.

### TGF-β2 induces autophagy in human glioma cell lines in a time and dose-dependent manner

To investigate the exact relationship between TGF-β2 and LC3B in glioma, we treated the tumor cells with a TGF-β2 dose gradient ranging from 0.1 ng/ml to 10 ng/ml, and after 24 h, Western blotting was used to detect autophagy levels. As an increase in the LC3B-II/I ratio is a credible marker of autophagy enhancement [30], TGF-β2 promoted endogenous LC3B-I to LC3B-II conversion in three different cell lines and one primary cell line in a dose-dependent manner (Fig. 2a Additional file 6: Figure S6a). To determine the proper time required for TGF-β stimulation, we set a gradient time course and also tested the conversion ratio by western blot. Our results indicated that 24 h was appropriate to induce glioma autophagy (Fig. 2b and Additional file 6: Figure 6b).

**Fig. 2:** TGF-β2 promotes LC3 conversion with time- and dose-dependent effects. **a** Immunoblot analysis showed the dose-dependent effect of TGF-β2 treatment (24 h) on the endogenous conversion of LC3 in U251, T98 and U87 cell lines. The LC3B-II/I ratio (middle) was calculated using ImageJ 1.36b. **b** Time-dependent effects of (10 ng/ml) on U251, T98 and U87 cell lines. **c** U251, T98, and U87 cells stably that expressed GFP-LC3B from lentiviruses after TGF-β2 treatment was observed by fluorescence microscopy. The percentage of positive cells were quantified (scale bars 50 μm). **d** Transmission electron microscopy showed the formation of autophagosomes after TGF-β2 treatment (10 ng/ml, 24 h) in U251 cells. Bottom left, enlarged image. Representative images of autophagosomes are shown at the bottom (arrows). The number of autophagosomes per cell were quantified. **e** In primary cells, TGF-β2 could also initiate autophagy showed by western blot under the same condition of cell lines’ (10 ng/ml, 24 h). **f** TGF-β2-induced autophagy are not affected upon mTOR agonist 3-MA (25 ng/ml). And blocking the autolysosomal step of autophagy by Baf (10 ng/ml) showed up-regulation of SQSTEM/P62. Graph shows densitometric analysis of P62 and actin expressed as p62/actin ratio. **g** Microarray analysis showed autophagy-related gene expression levels in TGF-β2-treated U251 cell lines. (Student’s t-test; Columns, means of triplicate assays, **, *P* < 0.01; error bars are SD)

To confirm this phenomenon, we applied a lentiviral system and generated stably expressing GFP-LC3 cells to monitor autophagy (TGF-β2, 10 ng/ml, 24 h) (Fig. 2c). In autophagy studies, the analysis of GFP-LC3 localization is widely performed by counting LC3-GFP positive cells (LC3-GFP dots greater than four) [30]. We found that TGF-β2 treatment increased the percentage of LC3-GFP positive cells (Fig. 2c). As transmission electron microscopy is the gold standard for identifying autophagosome double-membrane structure, we used transmission electron microscopy and found that glioma autophagosomes increased after TGF-β2 treatment (Fig. 2d, Additional file 2: Figure S2a).

Considering the disadvantage of cell lines to represent glioma’s characters, we introduced primary cells in our in vitro experiment, which were obtained from newly surgical GBM samples in Qilu hospital and grades were confirmed by pathology IHC. As shown in western blot (Fig. 2e), TGF-β2 could also initiate autophagy in primary cell under the same condition (10 ng/ml; 24 h) which indicate that the results of cell lines may represent the primary cells to some extent in our experiment.

Effects of 3-MA or Baf on autophagy flux mediated by TGF-β were also determined. Glioma cells were incubated with 3-MA (10 mmol/L) or Baf (10 nmol/L) during the treatment with TGF-β2 (Fig. 2f) and results indicated that Baf could effectively inhibit TGF-β induced autophagy except for 3-MA. According to the results of a microarray that compared the control and TGF-β2 treatment groups, the mRNA levels of the autophagy related genes BECN1, ATG5, ATG7 were also up-regulated after TGF-β2 treatment (Fig. 2g). To summarize, autophagy can be induced by TGF-β2 (10 ng/ml, 24 h) and blocked by Baf (10 nmol/L, 24 h). We next investigated the biological significance of this phenomenon.

### TGF-β2 induced autophagy is related to glioma invasion and migration

To explore the biological meaning of TGF-β2-induced autophagy in oncogenesis, we first introduced a stable siRNA expression system targeting the essential autophagy gene ATG5 and ATG7. Efficiency of siRNA was examined by Western blot (Fig. 3a), and the ratio of LC3B-I to LC3B-II conversion and SQSTM1 (also well known as P62) degradation indicated that siATG5, siATG7 was an effective target for inhibiting autophagy flux. As we know from previous studies, TGF-β2 promotes glioma oncogenesis behavior [9, 31, 32]. We used methods involving CCK-8 and BrdU proliferation assays to assess cell proliferation and observed no obvious effect after TGF-β2 treatment in normal tumor cells (NTC) or autophagy-deficient tumor cells (Fig. 3b, Additional file 3: Figure S3).

**Fig. 3:** Inhibition of autophagy impairs glioma invasive behavior initiated by TGF-β2. **a** Representative Western blots of SQSTM1 and LC3 conversion assays to evaluate the efficiency of siATG5 and siATG7 in tumor cells. **b** Brdu proliferation assays were performed on control tumor cells (U251, T98, and U87) and siATG5, siATG7 tumor cells after TGF-β2 treatement. Images were captured by fluorescence microscopy (scale bars, 50 μm) after 24 h and Brdu/DAPI ratio were calculated per fields in three independent assays. **c** Wound healing assay were also conducted with same conditions. Phase-contrast images (scar bars, 100 μm) were acquired at 1, 6, 12, 24, 36 and 48 h after scratching. The corresponding data relative from 1 to 48 h are expressed in the graph. **d** Eosin-stained sections of the Matrigel matrix. The average number of invading siATG5, siATG7 cells and NTC in four representative eosin-stained images (scale bars, 100 μm) were counted after 24 h of invasion (Student’s t-test; Scale bars are 100 μm, and columns, means of triplicate assays, *, *P* < 0.05; **, *P* < 0.01, ***, *P* < 0.001; error bars are SD)

Then we turned to examine the behavior of autophagy in glioma invasion and analyzed results with wound healing assays in U251, T98, and U87 cell lines. In stable siATG5 and siATG7 tumor cells, autophagy impaired groups exhibited delayed wound closure compared to scramble group tumor cells when exposed to TGF-β2 stimulation (Fig. 3c). And also we carried out a Transwell assay and found that fewer siATG5 and siATG7 cells migrated through the Transwell chamber micropores after TGF-β2 stimulation (Fig. 3d, Additional file 2: Figure S2b). Inefficient ECM degradation usually indicates potential changes in the function or expression level of matrix metalloproteinase (MMPs), which are involved in ECM degradation and the epithelial-mesenchymal transition (EMT). Summarizing the results above, TGF-β2 induced glioma autophagy participated in the invasive process but not tumor proliferation.

### TGF-β2 induced EMT in glioma cells could be blocked by suppressing autophagy

To identify the mechanism of autophagy-influenced glioma invasion, we conducted qRT-PCR to determine the expression levels of MMPs in normal glioma cells and Baf-treated tumor cells with or without TGF-β2 stimulation (Fig. 4a). The Baf treatment down-regulated the mRNA expression of the mostly MMP family in cells exposed to TGF-β2, and in contrast control group with TGF-β2 showed increasing expression levels of most MMPs (Fig. 4a, Additional file 4: Figure S4). MMP2 and MMP9, which are the most well-known MMPs for their important roles in tumor cell invasion [33, 34], were also down-regulated by Baf. And this finding was confirmed by Western blot experiments used to detect the cleaved, active forms of MMP2 and MMP9 (Fig. 4b). As the proteolytic cleavage of the ECM is usually governed by cell surface and soluble MMPs, we used an ELISA assay to detect soluble MMP2 and MMP9 in the supernatant of cultured NTC- and Baf-treated cells, similar results were expressed (Fig. 4c). In addition to degrading ECM, MMP2, 9 are also markers of EMT. We used Western blotting to examine other EMT markers to assess the potential association between EMT, TGF-β2 and autophagy. N-cadherin, Vimentin, Slug2, and β-catenin increased in normal tumor cells (NTC) treated with TGF-β2 but decreased in autophagy-inhibited cells however E-cadherin showed reverse effect (Fig. 4d). Immunofluorescence again demonstrated a direct change of Vimentin and N-cadherin between NTC and Baf-treated cells after treatment with TGF-β2 (Fig. 4e, f). Taken together, these results provide a potential explanation for how autophagy impairs glioma invasion: the inhibition of autophagy may lead to an impaired EMT and a failure in the invasive behavior of glioma cells.

**Fig. 4:** Impairing autophagy inhibits MMP generation and secretion as well as EMT-like process, which lead to deficient glioma invasion. **a** mRNA expression levels of MMP family genes (MMP1–3, 7–9, 11–17) in U251, T98, and U87 NTC and Baf-treated cells with TGF-β. **b** Immunoblot analysis showing the effects of Baf on MMP2, MMP9, and MMP14 synthesis in glioma cell lines after exposed to TGF-β2. **c** The MMP2 and MMP9 secretion levels in supernate obtained from NTC and Baf-treated cells were tested using an ELISA kit. **d** The expression levels of EMT markers (N-cadherin, E-cadherin, Vimentin, β-catenin, and Slug2) in different groups were tested by Western blots. **e**, **f** Immunofluorescences observed N-cadherin and Vimentin expression in glioma cell lines after treated with TGF-β2 and Baf, Representative images of three independent experiments are shown (scale bars, 50 μm). (Student’s t-test; Columns, means of triplicate assays. Bars, SD. **, *P* < 0.01; ***, *P* < 0.001)

### Autophagy induction by TGF-β2 is mediated by c-Jun NH2-terminal kinase and the Smad pathway and in turn affects TGF-β2 synthesis and secretion

We next investigated the exact mechanism of the process. Because autophagy is usually activated through mTOR-dependent and mTOR-independent pathways [35, 36], we used Western blotting to determine whether either of these pathways functioned in this process. Inhibiting the AKT-PI3K-mTOR pathway by 3-MA did not attenuate TGF-β2-induced autophagy (Fig. 5a). Thus, we assessed the mTOR-independent pathway using the c-Jun NH2-terminal kinase (JNK) pathway inhibitor SP600125. This treatment efficiently down-regulated the LC3B-II level in TGF-β2 treated glioma cells, indicating JNK pathway was one potential pathway responsible for TGF-β2 induced autophagy. TGF-β signals also went through downstream Smad and non-Smad pathways. The JNK pathway is a non-Smad pathway, and therefore we examined whether the Smad pathway also participated in autophagy induction. After transient siRNA with siSmad2, the addition of TGF-β2 did not stimulate autophagy in glioma, suggesting that the Smad pathway was also involved in autophagy induction (Fig. 5b).

**Fig. 5:** TGF-β2 activates glioma autophagy via Smad dependent and independent pathways, which in turn promote TGF-β autocrine signaling and boost glioma invasion. **a** The effects of PI3K kinase inhibitor 3-MA (10 μmol/L) and the JNK pathway inhibitor SP600125 (10 μmol/L) on TGF-β induced autophagy. **b** Immunoblots showed autophagy was attenuated in siSmad2-treated tumor cells though treated with TGF-β2. **c** Results showed level of TGF-β2 autocrine loop after promoting or inhibiting autophagy with Rapamycine or siATG5. **d** ELISA verified TGF-β2 level change after glioma cells treated with rapamycin and ATG5 knock down. **e** Quantitative reverse transcription-PCR analyses about Smad2, Smad3 and Smad7 which were compared between glioma cells treated with rapamycin, CQ and the TGF-β2 inhibitor LY2157299. **f** Immunoblots showed that inhibiting the TGF-β pathway with LY2157299 may cause an inefficient EMT. **g** The combination of CQ and LY2157299 inhibited autocrine TGF-β2 signaling in glioma cells. **h** ELISA results showed that siSmad2- and siATG5-treated tumor cells exhibited low L-lactate levels after TGF-β2 treatment. **i**, **j** L-lactate promoted glioma EMT marker expression and can be inhibited by CQ. (Student’s t-test; Columns, means of triplicate assays. Bars, SD. *, *P* < 0.05; **, *P* < 0.01; ***, *P* < 0.001)

Based on previous study, TGF-β2 function requires sustained autocrine signaling by tumor cells [31]. Thus, we explored whether autophagy would in turn affect TGF-β2 autocrine signaling (Fig. 5c), finding that rapamycin elevated the endogenous TGF-β2 levels in glioma cell and enhanced Smad2 phosphorylation. However, in siATG5-treated tumor cells, the Western blotting results showed reverse effect (Fig. 5c). The ELISA assay for TGF-β2 also demonstrated these phenomenon (Fig. 5d).

We next explored how autophagy influenced TGF-β2. The qRT-PCR results demonstrated that enhancing autophagy by rapamycin increased the R-Smad expression levels (Smad2, Smad3) and decreased the I-Smad expression level (Smad7). In contrast, CQ down-regulated Smad2 and Smad3 and up-regulated Smad7 (Fig. 5e). Microarray also indicated that promoting autophagy could also in turn regulate TGF-β genes’ expression (Fig. 5f). LY21457299 is a clinical applied TGF-β inhibitors, however Western blotting demonstrated that LY2157299 had little effect on the endogenous TGF-β2 levels. After blocking autophagy flux with CQ or siATG5, the TGF-β2 level decreased (Fig. 5g).

Lactate was also reported to promote TGF-β synthesis and MMP2 production in glioma cells [37]. And lactate was associated with autophagy process tightly. We hypothesis that autophagy may mediate TGF-β2 autocrine via lactate secretion. In our experiments, lactate synthesis was increased in TGF-β2-stimulated tumor cells however decreased after siATG5 or CQ-treatment (Fig. 5h). And when we added exogenous lactate in cultured tumor cells, results confirmed that lactate could stimulate TGF-β2 and MMP2 expression and EMT-related protein changes, however CQ, except for LY2157299, could inhibit this process (Fig. 5i). Therefore, we summarized that TGF-β2 could induced autophagy in glioma via both Smad and non-Smad pathway (JNK pathway), and inhibiting autophagy could also in turn mediated endogenous TGF-β2 level in an autocrine fashion which might resulted from the changing of lactate level secreted by glioma cells.

### TGF-β2 and autophagy mediated energy mitochondria function of glioma

In addition to the signal pathway activation and invasion related genes variation, there might be other mechanisms leading to the failure of TGF-β2 caused by autophagy inhibition. As tumor cell invasion is a highly energy- and material-consuming process [23, 24] and autophagy is tightly associated with tumor metabolism [26, 38, 39], We thus hypothesized that TGF-β2-induced autophagy is enhanced to generate more ATP and materials for invasion. First we introduced the MitoTracker Red probe to observe the mitochondrial morphology and localization. Based on one newly issued research [40], we identified the mitochondria morphology as fragmented, intermediate and tubular according to the length of the mitochondria (Fig. 6a, Additional file 4: Figure S4a). In our experiment, tubular form was found to be a more favorable form in the cell invasion apex and underwent more trafficking. TGF-β2-treated NTCs favored the tubular mitochondria, whereas autophagy inhibited tumor cells formed more fragmented mitochondria.

**Fig. 6:** TGF-β2 and autophagy-mediated energy generation of glioma and mitochondria function. **a** Control or autophagy inhibited tumor groups with or without TGF-β2 treatment (10 ng/ml, 24 h) were stained with MitoTracker Red and classified as three forms (Scale bars, 50 μm). Percentages of the different morphologies were assessed. **b** Mitochondria trafficking capacity were divided by the distance from the mitochondria to nuclei visualized by MitoTracker Red and then were classified shown by the representative images (scale bars, 50 μm). Percentages were also calculated. **c** JC-1 probe was added to NTC and Baf-treated tumor cells with or without added TGF-β2 to test the mitochondrial membrane potential (△Ψm). **d** The quantitative analysis of △Ψm was conducted by flow cytometry (one-way ANOVA, columns: percentage of low △Ψm cells). **e** Immunoblots presented mitochondria fussion/fission related markers affected by TGF-β and Baf (Student’s t-test; Columns, ratio of P-Drp1/Drp1. Bars, SD. *, *P* < 0.05; **, *P* < 0.01). **f** OCR and ECAR in normal and autophagy cells inhibited with or without TGF-β2 treatment. OCR and ECAR were measured using the XF24 Seahorse Analyzer. **g**, **h** ATP and L-lactate levels were significantly increased upon treatment with TGF-β2.and baf treatment attenuated this effect, as examined using an ATP and L-lactate kit assay (Student’s t-test; Columns, means of triplicate assays. Bars, SD. *, *P* < 0.05; ***, *P* < 0.001)

Mitochondrial trafficking can also be classified as three forms [41]: perinuclear, polarized and infiltrating (Fig. 6b, Additional file 5: Figure S5a) according to the distance from nuclei to mitochondria. Then TGF-β group showed an increased percentage of the polarized form and Baf group showed more perinuclear form (one-way ANOVA, polarized form, U251 Con 40 ± 2.1% vs TGF 72 ± 6.2% vs Baf 30 ± 5.5% *p* = 0.019, perinuclei Con 52 ± 3.7% vs TGF 20 ± 4.8% vs Baf 65 ± 6.2% *p* = 0.026). That indicated Baf stopped TGF-β2 stimulation reprogramming mitochondrial trafficking to fuel tumor cell invasion at a long distance (Fig. 6b).

Apart from above two factors, mitochondrial membrane potential (△Ψm) is also a vital factor for ATP generation. We used a JC-1 probe to detect the changes of △Ψm in mitochondria. JC-1 probe is an ideal probe that forms J-aggregates with red fluorescence in high △Ψm conditions and J-monomers with green fluorescence in low △Ψm conditions [42]. We observed red fluorescence increasing after TGF-β2 treatment in NTCs and green fluorescence enhancing in Baf treatment tumor cells though also treated with TGF-β2 (Fig. 6c, Additional file 5: Figure S5b). This phenomenon was confirmed by flow cytometry (FCM): one-way ANOVA, green percentage, U251 Con 4.55 ± 3.26% vs TGF 1.82 ± 0.67% vs Baf 15.55 ± 3.28% *p* = 0.038 (Fig. 6d).

As we could observe the changes of mito-fussion and fission in TGF-β2 and Baf treated groups, the exact molecular signal pathway were also explored by Western blot according to related studies [40, 43]. Results indicated that the phosphorylation of Drp1 and the expression of Opa3 and Mitofusion1 was responsible for the effect (Fig. 6e).

Besides the mitochondria changing, tumor cells were also characterized for aerobic glycolysis (Warburg-like metabolism). We thus recurred to XFe24 analysis (Seahorse) and found that TGF-β2 also altered metabolism program towards to aerobic glycolysis which resulted in a higher consumption rate of oxygen (OCAR) and an increased extracellular acidification (ECAR) to sustain ATP providing and then inhibiting autophagy could block this process (Fig. 6f). ATP assay kit and L-lactate testing kit also confirmed the same results (Fig. 6g, h). These results above provided a further explanation for how inhibiting autophagy might impair TGF-β2-stimulated glioma invasion: the mitochondria relocalization, morphological changes, down regulation in membrane potential and aerobic glycolysis reprogramming.

### In vivo xenograft models demonstrated that treatment with combined TGF-β2 and autophagy inhibition provides more benefits than galunisertib single application

We used tumor xenograft models to test this finding and explore the clinical significance. After planting U87 cells in severe combined immune deficiency (SCID) mice, we assigned the animals to the following treatment groups: PBS group, LY2157299 group, CQ group and LY2157299 combined with CQ group. LY2157299 combined with CQ was the most favorable treatment for the mice with tumor xenografts according to the survival time and tumor volumes results monitored by 3 Tesla MRI (Fig. 7a, b), while groups with single CQ showed limited cure effect on tumors which was also in accord with other reference [44]. After 50 days, samples were obtained from the SCID mice and stained with HE, images showed that brains of groups with PBS was infiltrated with tumor cells among the normal brain and tumors borders, while combination treatment with LY2157299 and CQ showed sharp and clear borders between normal tissues and tumor (Fig. 7c). This may indicated a more moderate invasiveness in dual-drug used groups. With IHC, we could also observed a decreased expression level of TGF-β in LY2157299 treated groups (*P* = 0.0476) and combination drugs groups showed the least expression level (*P* = 0.0056) (Fig. 7d).The in vivo results showed the potential benefits of combined treatment using TGF-β and autophagy pathway inhibitors as CQ could improve the effect of TGF-β inhibitors. This finding provides additional evidence that TGF-β may partially act via autophagy to function in glioma invasion.

**Fig. 7:** LY2157299 combined with CQ improved the outcome of glioma compared to treatment with only LY2157299 or CQ in vivo. **a** In vivo experiments show that the combination of LY2157299 (75 mg/kg/d) and CQ (25 mg/kg/d) had better capacity to inhibit glioma invasive behavior and proliferation monitored and measured by 3T MRI. **b** Tumor volume monitored by MRI and calculated, results showed that the combination group got the smallest tumor volume than single LY2157299 group and control group (Student’s t-test; Columns, means of triplicate assays. Bars, SD. *, *P* < 0.05; ***, *P* < 0.001). **c** Log-rank (Mantel-Cox) test demonstrated the LY2157299/CQ group brought a longer survival time compared to LY2157299 group (P=0.02). **d** H&E staining of PBS, LY2157299 and LY2157299/CQ groups, and dual-drug treatment group showed a more sharp-edged and clear tumor borders as well as less tumor infiltrating and invasion (N, normal brain tissue; T, tumors in brain, scale bars, 100μm). **e** Immunochemistry (IHC) showed more LC3B and TGF-β2 positive cells in control groups and less LC3B positive cells in LY2157299 groups and the least TGF-β2 positive cells in dual-drug used groups (scale bars, 50μm). IRS model quantatively analyzed LC3B and TGF-β2 expression levels in IHC (Wilcoxon matched-pair test: Bars, SD. **, *P* < 0.01)

## Discussion

In the present study, we explored one finding that TGF-β2 was highly expressed and correlated with LC3B in clinical samples. And in vitro, TGF-β2 induced autophagy in glioma cell lines in a time- and dose-dependent fashion. As TGF-β is an abundant component of the glioma tumor microenvironment, our research may provide another explanation as to why high levels of LC3B expression are usually found in high grade gliomas. In addition to hypoxia and starvation, TGF-β2 and other cytokines (IL-2, IL-6, TNF-α, IFN-γ) may potentially promote glioma autophagy. Much research has been focused on cytokines and autophagy [45, 46], however few answered the question that what was the meaning of cytokine-initiated autophagy.

Our study demonstrated that autophagy flux is vital for TGF-β-induced glioma invasion and we attributed partial reasons to the failure of EMT, which should increase with TGF-β2 stimulation. Reasonablely illustration in our study was that autophagy blockage suppressed EMT-related protein expression and also decreased the level of L-lactate which induces TGF-β2 autocrine and promotes EMT marker expression. Moreover, other researchers have also reported that autophagy-related genes such as BECN1 and SQSTM1 are associated with EMT [47, 48]. These findings provide a new opportunity for discussing the EMT under autophagy during tumor invasion. However, the exact mechanism by which autophagy influences the EMT is mysterious, and further exploration needs to be done in the future.

In addition to EMT, autophagy and TGF-β are both broadly involved in tumor metabolism. Tumor invasion is a high-energy-consumption process, so the ATP generation failure induced by autophagy inhibition may also explain the deficiencies in tumor invasion (Fig. 6g, h). Here is our hypothesis that tumor cells evolved to allow TGF-β to activate autophagy as TGF-β boosted metabolism as well as large reactive oxygen species (ROS) production [49] and if there was no factor eliminating ROS promptly, tumor cells would soon apoptosis for mitochondria damage. Besides, there was a long debate about mitochondrial fusion and fission, including which process is more favorable for tumor invasion and metabolism. Interestingly, TGF-β promotes glioma invasion and elevates ATP generation, causing increased fusion forms of mitochondria. Although we have determined some proteins (Drp1, Opa3 and Mitofusion1) of mitochondira conversion which TGF-β targeted on, a lot of work still need to be done to enrich the outline of the process. Autophagy may have a larger role in tumor invasion that has yet not to be determined.

The two main downstream pathways of TGF-β signaling are the Smad-dependent and Smad-independent pathways [31, 50]. In our study, both were found to participate in TGF-β2-induced autophagy in glioma (Fig. 5a, c). TGF-β activates the PI3K-Akt-mTOR pathway during the TGF-β-induced EMT, however the phosphorylation of mTOR usually inhibits autophagy. TGF-β may play both stimulatory and inhibitory roles in autophagy. But at least in U251 cells, the autophagy stimulation by the Smad and JNK pathways may outweigh the antiautophagic effect of mTOR. Whether this change from an inhibitory role to a stimulatory role in autophagy indicates that the TGF-β changes from functioning as a tumor suppressor to tumor promoter also needs more exploration.

We knew that the TGF-β effects on glioma require sustained autocrine pathway activation [31]. Therefore, we explored the effect of autophagy flux in cytokines’ autocrine loop. Our results demonstrated that autophagy inhibitors mediated TGF-β expression in mRNA levels (Fig. 5e). Experiments (Fig. 5h) also proved that the increased amounts of metabolic products resulting from enhanced autophagy (lactate) leads to increased autocrine TGF-β2 levels. According to these results, TGF-β pathway might influence the invasive behaviors of tumor cells via TGF-β-autophagy-lactate-TGF-β loop. LY2157299 was a newly identified TβRI inhibitor with phase III clinical trials. However, in glioma LY2157299 showed little effect on the TGF-β2 autocrine level, which may result in keeping the tumor cells in a favorable microenvironment that tends to promote oncogenesis. Thus, we advised to administer a combined treatment of LY2157299 and CQ to mice, based on the tumor xenograft models results.

In clinical trials, it is still controversial that LC3B is associated with the grade of the glioma. High LC3B expression of LC3B sometimes is associated with an improved outcome for patients with poorer performance. For patients with normal performance, survival was better for patients with lower LC3B staining [51]. We found that TGF-β2 and LC3B dual positive patients had distinctly shorter survival times than TGF-β2 positive and LC3B negative patients. We hypothesize that the autophagy level may be a valid predictor of patient prognosis only in patients whose IHC showed both TGF-β2 and LC3B staining. Many factors can influence autophagy, and possibly only when autophagy was mainly activated by cytokines rather than other factors, autophagy was an effective predictor. Another explanation is that TGF-β2 only induces glioma autophagy when it reaches a certain level in the tumor microenvironment. Therefore, LC3B positive staining usually indicates a higher level of TGF-β2 in glioma, leading to a poor outcome. These hypotheses was verified primarily with statistical results. However, whether other cytokines are coordinated with these results and whether this could be a widely used phenomenon remain interesting, unanswered questions.

Overall, our work provides a novel role for autophagy in TGF-β2-induced glioma invasion that potentially occurs through the regulation of energy metabolism and autocrine TGF-β (mode pattern Additional file 7: Figure S7). The functional alteration of TGF-β from a tumor suppressor to a tumor promoter may be associated with autophagy. Furthermore, the combination of TGF-β and autophagy inhibitors improves disease in vivo, which may in turn guide the application of CQ in clinical cases. More generally, this study resulted in a systematic identification of cytokines and autophagy, which can also be used for similar studies.

## Conclusion

Our findings elucidated a potential mechanism of autophagy-associated glioma invasion that TGF-β2 could initiate autophagy via Smad and non-Smad pathway to promote glioma cells’ invasion. During this process, the alteration of epithelial-mesenchymal transition and metabolism conversion were considered to involved in. And based on this study, we believe a new approche to cure glioma could be found and new opinion could be inspired to refresh our view about cancer.

## Additional files

Additional file 1: Figure S1. The human primers used in Fig. 4a were listed in this supplementary figure. (TIFF 2375 kb)

Additional file 2: Figure S2. **a** the results of TEM in other two cell lines (U87 and T98) showing the similar phenomenon with U251. **b** the results of woud healing in other two cell lines (U87 and T98) showing the similar phenomenon with U251. (TIFF 3664 kb)

Additional file 3: Figure S3. CCK-8 assasy was performed to assess cell viability in U251, T98, U87 cells. Columns, means of triplicate assays. Bars, SD; (TIFF 1016 kb)

Additional file 4: Figure S4. The exact value of qPRC test in Figure 4a, and resutls were caculated by t-test. (TIFF 1768 kb)

Additional file 5: Figure S5. The figures of mitotracker and JC-1 probe in other two cell lines (U87 and T98) showing the similar phenomenon with U251. (TIFF 5335 kb)

Additional file 6: Figure S6. ImageJ was introduced to assess the western blot results in in Fig. 2a & b in U251, T98, U87 cells. Columns, means of triplicate assays. Bars, SD; (TIFF 1261 kb)

Additional file 7: Figure S7. Modern pattern of the whole research showing that autophagy-associated glioma invasion that TGF-β2 could initiate autophagy via Smad and non-Smad pathway to promote glioma cells’ invasion. (TIFF 1134 kb)

## Abbreviations

AA: Astrocytoma
Baf: Bafilomycin A1
CQ: Chloroquine
DMSO: Dimethyl sulfoxide
EMT: Epithelial-mesenchymal transition
GBM: Glioblastoma multiforme
JNK: c-Jun NH2-terminal kinase
mTOR: Mammalian target of rapamycin
NTC: Normal tumor cell
Rapa: Rapamycin
